RETRACTED

# Heme Oxygenase-1 Inhibits the Proliferation of Hepatic Stellate Cells by Activating PPAR*γ* and Suppressing NF-*κ*B

**DOI:** 10.1155/2022/8920861

**Published:** 2022-01-10

**Authors:** Hui Yang, Li Zhang, Jie Chen, Xiaoqian Zhang, Zhongfu Zhao, Longfeng Zhao

**Affiliations:** ^1^Department of Infectious Diseases, The First Hospital of Shanxi Medical University, Taiyuan, Shanxi Province, China; ^2^Institute of Hepatopathy, Changzhi Medical College, Changzhi, Shanxi Province, China

## Abstract

**Background:**

Hepatic stellate cells (HSCs) are reported to play significant roles in the development of liver fibrosis. Heme oxygenase-1 (HO-1) is a key rate-limiting enzyme, which could decrease collagen synthesis and liver damage. Nevertheless, it was yet elusive towards the function and mechanism of HO-1.

**Methods:**

An HO-1 inducer Hemin or an HO-1 inhibitor ZnPP-IX was used to treat the activated HSC-T6, respectively. MTT assay was adopted to detect cell proliferation. Immunocytochemical staining was employed to test the levels of alpha-smooth muscle actin (*α*-SMA), peroxisome proliferator-activated receptor-*γ* (PPAR*γ*), and nuclear factor-kappa B (NF-kappa B) levels in HSC-T6. HO-1, PPAR*γ*, and NF-*κ*B expression levels were measured by qRT-PCR and Western blotting. ELISA was then used to detect the levels of transforming growth factor- (TGF-) beta 1 (TGF-*β*1), interleukin-6 (IL-6), serum hyaluronic acid (HA), and serum type III procollagen aminopeptide (PIIIP).

**Results:**

HSC-T6 proliferation was inhibited in Hemin-treated HSCs. The levels of *α*-SMA, HA, and PIIIP and the production of ECM were lower in Hemin-treated HSCs, whereas those could be rescued by ZnPP-IX. NF-*κ*B activation was decreased, but PPAR*γ* expression was increased after HO-1 upregulation. Furthermore, the levels of TGF-*β*1 and IL-6, which were downstream of activated NF-*κ*B in HSC-T6, were reduced. The PPAR-specific inhibitor GW9662 could block those mentioned effects.

**Conclusions:**

Our data demonstrated that HO-1 induction could inhibit HSC proliferation and activation by regulating PPAR*γ* expression and NF-*κ*B activation directly or indirectly, which makes it a promising therapeutic target for liver fibrosis.

## 1. Introduction

Hepatic stellate cells (HSCs) are reported to play significant roles in liver fibrosis progression. The HSCs undergo a transition from quiescent cells into active cells during liver injury, which is the principal source of the extracellular matrix (ECM). Therefore, preventing the proliferation and activation of HSCs is an effective strategy to reverse liver fibrosis.

Nuclear factor-kappa B (NF-*κ*B), a crucial nuclear transcription factor, can medicate the expression of various inflammation-related proteins, including tumor necrosis factor-*α* (TNF-*α*) and interleukin-1 (IL-1). NF-*κ*B is associated with the phenotype of the HSCs. Activated NF-*κ*B promotes the proliferation and ECM production of HSC, which is significant in the process of liver fibrosis [1]. The peroxisome proliferator-activated receptor (PPAR), a ligand-activated nuclear receptor, exists widely in the organism and has three isoforms: *α*, *β*, and *γ*. PPAR*γ* expressed in HSCs is beneficial for maintaining the HSCs' static phenotype [2]. PPAR*γ* upregulation leads to a significant decrease in HSC activation and reverses the progression of liver fibrosis. PPAR*γ* could directly combine with the p50/p65 subunit of NF-*κ*B to form a transcriptionally inhibited complex, which could decrease the binding activity of NF-*κ*B and inhibit DNA synthesis of NF-*κ*B, thus inhibiting its expression [3]. PPAR*γ* could also inhibit NF-*κ*B transcription by competitively combining with the coactivating factors CREB-binding protein (CBP) and P300 and could then induce HSC apoptosis [4].

RETRACTED

Heme oxygenase-1 (HO-1), as a rate-limiting enzyme, degrades the heme into iron, biliverdin, and carbon monoxide, which share antioxidative, anti-inflammatory, and antiapoptotic activities [5]. Increasing evidence supports that HO-1 can protect liver cells from damage caused by multiple causes, such as acute liver injury and liver transplantation [6]. Studies have shown that the HO-1 promoter region contains binding sites of NF-*κ*B; therefore, HO-1 activity is directly related to NF-*κ*B [7]. HO-1 can inhibit NF-*κ*B expression in macrophages [8]. In addition, a study found that there was crosstalk between HO-1 and PPAR [9]. Gene polymorphisms in the HO-1 promoter region have effects on the transcriptional activity of PPAR subtypes [10]. The inhibitory effect of cell proliferation induced by the PPAR ligand could be reversed by downregulating HO-1 activity. The HO-1-induced upregulation of PPAR could restrain the proliferation of pulmonary artery smooth muscle cells, which could be attenuated by a siRNA that knocks down HO-1 expression [11].

In the previous study, Du et al., have endeavored to investigate the relationship between HO-1 and nonalcoholic fatty liver disease (NAFLD) and demonstrated that the induction of HO-1 could eliminate steatohepatitis and hepatic fibrosis in the progression of NAFLD [6], thus substantiating a significant role of HO-1 against heme-mediated steatohepatitis-related liver fibrosis.

In our previous study, we have reported the role of HO-1 in carbon tetrachloride- (CCl_4_-) induced liver fibrosis [12]. Our data demonstrated that HO-1 induction could decrease collagen synthesis and the degree of fibrosis, thus preventing liver fibrosis progression. However, the precise effects of HO-1 on HSCs and the underlying mechanisms still remain unclear. Currently, there is also still limited evidence of HO-1 on HSC activation and pathogenesis. We hypothesized that HO-1 induction might affect HSC proliferation and activation and might decrease the release of inflammatory factors from HSCs, which might upregulate PPAR*γ* and suppress the NF-*κ*B pathways in HSCs.

RETRACTED

## 2. Materials and Methods

### 2.1. Materials and Chemicals

Dulbecco's modified Eagle's medium (DMEM) and fetal bovine serum (FBS) were purchased from Invitrogen (Carlsbad, CA, USA). Hemin (ferriprotoporphyrin IX, a potent inducer of HO-1 [13]) and zinc protoporphyrin IX (ZnPP-IX, a specific HO-1 antagonist [14]) were the products of Sigma (St. Louis, MO, USA) [15]. The final concentrations of Hemin and ZnPP-IX were both 0.5 mg/ml. The anti-HO-1 and anti-PPAR*γ* antibodies were obtained from Cell Signaling Technology (Danvers, MA, USA). The anti-phospho-NF-*κ*B p65 and anti-*α*-smooth muscle actin (*α*-SMA) antibodies were acquired from Santa Cruz Biotechnology (Santa Cruz, CA, USA). GW9662 and rosiglitazone were the products of Cayman Chemical (St. Louis, MO, USA) which were used as PPAR*γ*-specific antagonists and agonists, respectively.

### 2.2. Cell Culture and the Selection of the Drug Concentration

HSC-T6 were obtained from Dr. Zhongfu Zhao (Changzhi Medical College, Shanxi Province, China) and grown in DMEM containing 10% FBS at 37°C in a 5% CO_2_ incubator. HSC-T6 were used for experiments within 4-6 passages and incubated with various concentrations of Hemin (6.5, 13, and 26 *μ*g/ml) or ZnPP-IX (3, 6, and 12 *μ*g/ml) for 12, 24, and 48 hours. A lactate dehydrogenase (LDH) kit was used to determine the cytotoxicity of Hemin or ZnPP-IX [16]. The MTT assay kit was adopted for the analysis of cell viability based on the manufacturer's instructions. For the experiments described above, 13 *μ*g/ml Hemin and 6 *μ*g/ml ZnPP-IX were used for 24 hours; these doses were effective and innocuous in cells.

### 2.3. Cell Groups and Treatments

To determine the effects of HO-1 on HSC-T6 proliferation and activation, HSC-T6 were assigned into 4 groups. Cells in group A were cultured in normal sodium for 24 hours as a negative control. Cells exposed to 13 *μ*g/ml Hemin or 6 *μ*g/ml ZnPP-IX were, respectively, named group B and group C. Cells in group D were cultured with 13 *μ*g/ml Hemin and 3 *μ*g/ml ZnPP-IX. Furthermore, the HSC-T6 cells were divided into another 5 groups to evaluate the levels of PPAR*γ*, NF-*κ*B, and inflammatory factors. Except for the control group, cells in the Hemin-treated group and the ZnPP-IX-treated group were added into the same dose of Hemin and ZnPP-IX as above. But cells in the Hemin+GW9662 cotreated group were challenged with 5 *μ*mol/l GW9662 for 30 minutes prior to Hemin. Cells in the ZnPP-IX+rosiglitazone cotreated group were exposed to 10 *μ*mol/l rosiglitazone for 30 minutes prior to ZnPP-IX.

RETRACTED

### 2.4. Immunostaining for *α*-SMA, PPAR*γ*, and NF-*κ*B

HSC-T6 cultured in 6-well plates containing sterile coverslips in each well were fixed with 4% polyoxymethylene for 30 minutes at 4°C. After 0.1% Triton X-100 permeabilization, cells were blocked with 10% normal goat serum and then probed with anti-*α*-SMA, anti-PPAR*γ*, or anti-NF-*κ*B. The slides were probed with the corresponding biotinylated or fluorescein isothiocyanate- (FITC-) labeled secondary antibodies for 30 minutes. The cells with the biotinylated avidin-biotin complex for 15 min were treated with 3,3′-diaminobenzidine for 5 minutes. Cells were then counterstained with the nuclear dye hematoxylin and were examined under the microscope. For the FITC-labeled cells, mount the coverslip on slides and observe through a fluorescence microscope. The images were analyzed and calculated using a computer program.

### 2.5. Quantitative Real-Time PCR for HO-1, *α*-SMA, PPAR*γ*, and NF-*κ*B Expression

Total RNA was isolated with an RNA TRIzol isolation reagent kit (Invitrogen, USA). A PrimeScript™ strand cDNA synthesis kit (Takara Biotechnology Co., Ltd.) was used for reverse cDNA reverse transcription. The PCR reactions were carried out using a PCR 7500 System and Power SYBR Green PCR Master Mix (Applied Biosystems; Thermo Fisher Scientific Inc.). The study includes the following primers: HO-1: (forward) 5′-CGTGCAGAGAATTCTGAGTTC-3′, (reverse) 5′-AGACGCTTTACGTAGTGCTG-3′; *α*-SMA: (forward) 5′-CTGAAGAGCATCCGACACTG-3′, (reverse) 5′-AGAGGCATAGAGGGACAGCA-3′; PPAR*γ*: (forward) 5′-TGTGGACCTCTCTGTGATGG-3′, (reverse) 5′-AGCTCTTGTGAACGGGATGT-3′; NF-*κ*B: (forward) 5′-AACACTGCCGAGCTCAAGAT-3′, (reverse) 5′-CATCGGCTTGAGAAAAGGAG-3′; and *β*-actin: (forward) 5′-GAGCTATGAGCTGCCTGACG-3′, (reverse) 5′-AGCACTTGCGGTCCACGATG-3′. Comparative quantification was determined with the 2-*ΔΔ*Cq method with *β*-actin used as the endogenous control [17].

### 2.6. Western Blotting

HSC-T6 were lysed by the RIPA buffer (Boster, China). After quantification of the protein concentrations with a Bicinchoninic Acid Protein kit (Beyotime, Shanghai, China), 40 *μ*g protein per lane was isolated on SDS-PAGE on a 12% gel and transferred onto PVDF membranes. Blots were then blocked with 5% nonfat milk and incubated with primary antibodies (4°C; overnight), followed by the incubation with HRP-conjugated secondary antibodies (1 h). Protein bands were developed with chemiluminescence detection reagents. The protein intensity was quantified with ImageJ.

RETRACTED

### 2.7. Enzyme-Linked Immunosorbent Assays (ELISA) for Measuring HA, PCIII, TGF-*β*1, and IL-6 Concentrations in the Cell Culture Medium

Supernatants of HSC-T6 were collected to detect the concentrations of HA, PCIII, TGF-*β*1, and IL-6 with ELISA kits (HopeYear Medical Products Co., Ltd., China). Each treatment was performed with five replicates.

### 2.8. Statistical Analysis

All data are expressed as means ± SD. Comparisons among multiple groups were analyzed using one-way ANOVA with the Newman–Keuls post hoc test, while the data in the two groups were compared by Student's *t*-test. *P* values < 0.05 were the standard used for statistical significance. All data analyses were performed with SPSS software (version 15.0).

## 3. Results

### 3.1. The Most Appropriate Concentrations and Incubation Periods for Hemin and ZnPP-IX

It was important to select the most effective concentrations and incubation periods for Hemin and ZnPP-IX to ensure the research was successful. The proliferation of HSC-T6 was reduced by Hemin in a concentration-dependent way beginning at 12 hours and was significant at 24 hours. ZnPP-IX also dose-dependently promoted HSC-T6 proliferation, which was significant at 24 hours (Figure 1(a)). The LDH kit was performed carefully to validate the cytotoxicity of Hemin or ZnPP-IX on HSC-T6. HSC-T6 incubated with 6.5 or 13 *μ*g/ml Hemin for 12 or 24 hours did not exhibit significant differences in LDH release but increased for 48 hours with 26 *μ*g/ml at all time points compared to the controls. In ZnPP-IX-treated cells, the LDH release was not significantly different compared to that in controls, with the exception of the group treated with 12 *μ*g/ml for 24 hours and all concentrations for 48 hours (Figure 1(b)). These results indicated that high concentrations of Hemin or ZnPP-IX and long incubation periods were toxic to cultured HSC-T6. Therefore, 13 *μ*g/ml Hemin and 6 *μ*g/ml ZnPP-IX were used to treat the cells for 24 hours in the subsequent experiments, which yielded optimal activity.

### 3.2. The Effects of Hemin or ZnPP-IX on HO-1 Expression and HSC Proliferation

The mRNA level of HO-1 in HSC-T6 was significantly increased in the Hemin group, while it decreased by 11.6% in the ZnPP-IX group. However, no significant differences were observed relative to the control (*P* = 0.504). However, HO-1 mRNA expression in the group exposed to Hemin and ZnPP-IX was still higher relative to that in the control and lower compared to that in the group treated with Hemin alone (Figure 2(a)). Western blot assay further supported the results of qRT-PCR (Figure 2(b)), which indicated that HO-1 expression in HSC-T6 was suppressed by ZnPP-IX and upregulated by Hemin, while the induction was partially reversed by a low concentration of ZnPP-IX.

RETRACTED

MTT assays further showed that HSC-T6 proliferation decreased by 16.15% in group B, which had higher levels of HO-1 expression induced by 13 *μ*g/ml Hemin, but increased by 12.28% in group C, which had low levels of HO-1 expression inhibited by 6 *μ*g/ml ZnPP-IX. In the group treated with 13 *μ*g/ml Hemin and 3 *μ*g/ml ZnPP-IX, HSC-T6 proliferation rebounded compared to that in the group treated with Hemin alone, but it was still notably elevated compared with that in the control (Figure 2(c)). The above data indicated that the induction of HO-1 expression could inhibit HSC proliferation, which could be reversed by the inhibition of HO-1.

### 3.3. Effects of HO-1 on the Levels of Activation Markers of HSCs

*α*-SMA and ECM overproduction are all important markers of HSC activation. After treating with Hemin, the expression of *α*-SMA decreased significantly but increased in the ZnPP-IX-treated group compared with the control (Figure 3(a)). Western blotting and qRT-PCR both confirmed that the *α*-SMA expression in the cotreated group was higher than that in the Hemin-treated group but less than that in the ZnPP-IX-treated group (Figure 3(b)). This result was further verified by *α*-SMA staining of cultured HSC-T6 (Figure 3(c)). HA and PCIII levels were found to be decreased in the Hemin group but significantly increased in the ZnPP-IX-treated group, similar to the results of *α*-SMA expression (Figure 4). These results indicated that the Hemin-induced HO-1 expression decreased *α*-SMA expression and HA and PCIII production in HSCs, while these effects could be reversed by ZnPP-IX.

### 3.4. Effects of HO-1 on PPAR*γ* Induction and NF-*κ*B Suppression in HSCs

Our previous research demonstrated that HO-1 might alleviate liver fibrosis and regulate the PPAR*γ* and NF-*κ*B expression in the liver by using the fibrosis rat model [12]. However, it is still unknown whether the effect described above is through HSC regulation. Therefore, we created a group where PPAR*γ* expression was inhibited before HO-1 induction and a group where PPAR*γ* expression was induced before HO-1 inhibition to observe the mRNA and protein levels of PPAR*γ* and NF-*κ*B in HSC-T6. Results reviewed that PPAR*γ* mRNA significantly increased and NF-*κ*B mRNA decreased in the Hemin-treated group compared to the control. While in the ZnPP-IX-treated group, PPAR*γ* mRNAs were reduced and NF-*κ*B mRNA increased (Figure 5(a)). We also found that HO-1 mRNA decreased by 19.6% and PPAR*γ* mRNA decreased by 27.3% in the group treated with GW9662 and Hemin relative to the group exposed to Hemin alone, but NF-*κ*B mRNA increased by 38.1%. HO-1 expression in this group decreased by 16.05% relative to that in the group only treated with Hemin. Moreover, PPAR*γ* expression decreased by 17.17%, while NF-*κ*B expression increased by 28.94%, which were consistent with those of their mRNAs (Figure 5(b)). Immunostaining analysis for PPAR*γ* and NF-*κ*B further verified these results (Figure 5(c)). These indicated that HO-1 was a key regulator involved in HSC activation through PPAR*γ* upregulation and NF-*κ*B inhibition; there was an interaction between HO-1 and PPAR*γ*, and the induction of HO-1 expression could directly or indirectly regulate NF-*κ*B activation through PPAR*γ* in HSCs.

RETRACTED

### 3.5. Effects of HO-1 on TGF-*β*1 and IL-6 Secretion from HSCs

To further verify the HO-1-mediated suppression of NF-*κ*B activation in HSCs, the secretion of TGF-*β*1 and IL-6 in HSC-T6 was detected, which are inflammatory factors that are downstream from activated NF-*κ*B. Both the levels of TGF-*β*1 and IL-6 were reduced in the Hemin-treated group when compared to the control, which was attenuated by pretreating with GW9662. However, the levels of TGF-*β*1 and IL-6 were elevated in the ZnPP-IX-treated group relative to other groups, which were also attenuated by pretreatment with rosiglitazone, although there was no significant difference in TGF-*β*1 secretion between the two groups (Figure 6). These demonstrated that the induction of HO-1 could restrain TGF-*β*1 and IL-6 secretion from HSCs, and the effects of HO-1 are associated with the levels of PPAR*γ*.

## 4. Discussion

HSC activation and proliferation are key events in liver fibrosis, which control the ECM deposition and the release of inflammatory factors. HO-1, an effective endogenous cytoprotective enzyme, can be induced in a variety of human and mammalian tissues to respond to various forms of oxidative stress and inflammatory damage. More and more evidence shows that inducing HO-1 expression is a crucial defense mechanism against multiple liver injuries [18–20]. Our recent studies in the CCl_4_-induced rat liver fibrosis model have suggested that the induction of HO-1 expression results in an apparent reduction in the *α*-SMA level, collagen synthesis, and liver damage, thereby preventing the progression of liver fibrosis. Although previous reports have strongly demonstrated that HO-1 has a protective role during the development of liver fibrosis, the molecular mechanism remains elusive. Actually, the animals' internal environment is complicated, and the results could have been impacted by other unavoidable factors. HSC-T6 which has been transfected with sarcoma virus 40 (SV40) has an activated phenotype in vitro [21]. In this experiment, HSC-T6 was used as a convenient model to investigate the mechanism of liver fibrosis, which could avoid the influence of the internal environment, and enabled us to detect the precise molecular mechanism of the protective effects of HO-1.

RETRACTED

To validate the positive and negative effects of HO-1 on HSCs, Hemin and ZnPP-IX were used as a specific agonist and inhibitor, respectively. In the present study, to clarify whether the induction of HO-1 could be attenuated by ZnPP-IX, a group that was exposed to the combination of Hemin and ZnPP-IX was designed, except for the groups exposed to Hemin or ZnPP-IX alone. We found that the rapid inhibition of HSC proliferation, *α*-SMA expression, and HA or PCIII secretion was accompanied by the upregulation of HO-1, which was partially reversed by ZnPP-IX. This evidence indicated that the effects of HO-1 were achieved by regulating HSC proliferation and activation during liver fibrosis progression.

PPAR*γ* and NF-*κ*B are two important nuclear transcription factors in the development of liver fibrosis. A previous study has reported that PPAR*γ* can maintain the quiescent phenotype of HSCs, which is closely related to liver fibrosis progression during hepatic injury [22]. PPAR*γ* can activate and upregulate Caspase-3 and Bax expression and can reduce Bcl-2 and NF-*κ*B expression to induce HSC apoptosis [23]. PPAR*γ* also can affect the signaling pathways that are correlated with HSC proliferation, activation, and apoptosis, particularly the NF-*κ*B pathway [24]. Therefore, we can prevent the progression of hepatic fibrosis by activating PPAR*γ* and then interfering with the NF-*κ*B pathway. Studies have shown that HO-1 and PPAR*γ* can regulate each other [9], and the HO-1 promoter region also has binding sites for NF-*κ*B. Our previous study has revealed that the variations of HO-1 in the rat liver were closely related to liver fibrosis development. HO-1 upregulation could inhibit liver fibrosis progression. It has also been shown that HO-1 inhibition or induction could affect PPAR*γ* and NF-*κ*B expression in the rat liver. Nevertheless, it is still unclear whether the liver-protective effect of HO-1 is related to HSCs. To further investigate the inhibition mechanism of HO-1 on HSCs, we analyzed the effect of HO-1 on PPAR*γ* and NF-*κ*B expression in HSC-T6 cells. Results described above indicated that Hemin-induced HO-1 expression dramatically increased PPAR*γ* expression and decreased NF-*κ*B expression in HSC-T6, which would prevent HSC proliferation and collagen production.

RETRACTED

To further investigate the effects of HO-1 on the expression of PPAR*γ* and NF-*κ*B, we designed the “Hemin+GW9662” group in the experiment, in which PPAR*γ* expression was inhibited by its specific inhibitor GW9662 before HO-1 induction. We also designed the “ZnPP-IX+rosiglitazone hydrochloride” group, in which PPAR*γ* was induced by its specific agonist rosiglitazone hydrochloride before HO-1 inhibition. Results revealed that HO-1 expression could be affected by PPAR*γ*, while PPAR*γ* and NF-*κ*B could regulate each other. In addition, our experiments also showed that smaller increases in HO-1 expression in HSC-T6 could cause an obvious reduction in NF-*κ*B expression. The amplifying effect of HO-1 might have occurred through direct regulation by NF-*κ*B combining with HO-1 promoter regions. However, HO-1 also could inhibit the NF-*κ*B signal transduction pathway by affecting PPAR*γ* expression and then inhibiting HSC proliferation and activation. Studies in other areas have shown that coregulation exists between HO-1 and PPAR*γ*. Our findings demonstrated that HO-1 could inhibit HSC proliferation and activation by not only directly upregulating PPAR*γ* expression or suppressing NF-*κ*B activity but also indirectly suppressing NF-*κ*B activity through PPAR*γ*. Yeh et al. [25] reported that HO-1 induction could mediate the effect of PPAR*γ* in suppressing the proliferation of rat pulmonary artery smooth muscle cells but that this effect was blocked by knockdown of HO-1 through siRNA transfection. Liu et al. [26] showed that HO-1 activation could attenuate the surge of inflammation-related cytokines and decrease the occurrence of cardiomyocyte apoptosis via inhibition of NF-*κ*B and activator protein 1 (AP-1) translocation. Lee et al. [27] indicated that upregulation of HO-1 could alleviate severe acute pancreatitis-associated lung injury in rats by decreasing NF-*κ*B activity drastically and inhibiting the serum levels of TNF-*α* and IL-6 significantly. Overexpression of HO-1 could protect against TNF-*α*-mediated airway inflammation by diminishing NF-*κ*B activation in both cultured human tracheal smooth muscle cells and mice.

Accumulating evidence suggests that PPAR*γ* could inhibit Smad3 phosphorylation and the transcription of Smad target genes, further inhibiting HSC proliferation, activation, and inflammatory cytokine and ECM release by blocking the TGF-*β*1/T R-I signaling pathway. Moreover, TGF-*β*1/connective tissue growth factor (CTGF) expression levels were significantly decreased [28]. It is noteworthy that the increased activation of NF-*κ*B in HSCs could further activate the levels of its downstream genes (IL-6, TNF-*α*, COX-2, ICAM-1, and others) to trigger or to aggravate inflammatory injury in the liver. TGF-*β*1 and other inflammatory cytokines further activate NF-*κ*B and increase HSC activation, eventually leading to liver fibrosis [29]. Therefore, the detection of TGF-*β*1 and IL-6 levels in HSCs could directly reflect HSC proliferation and activation and also reflect the levels of activated PPAR*γ* and NF-*κ*B in HSCs. In this study, TGF-*β*1 and IL-6 levels in each HSC-T6 group were detected after inhibiting or triggering HO-1 expression, which also verified the effect of HO-1 on HSC activation by regulating PPAR*γ* and NF-*κ*B. In this research, we found that upregulation of HO-1 could decrease the release of inflammatory factors from HSCs. This result was consistent with our previous animal experiment, which indicated that the HO-1 upregulation could attenuate the pathological and inflammatory changes in the liver. This study further demonstrated that TGF-*β*1 and IL-6 expression levels rebounded in the group pretreated with the PPAR*γ*-specific inhibitor GW9662 before Hemin compared to the group treated with Hemin alone. At the same time, TGF-*β*1 and IL-6 levels were decreased in the group pretreated with the PPAR*γ*-specific agonist rosiglitazone hydrochloride before ZnPP-IX compared to the group treated with ZnPP-IX alone. The changes in TGF-*β*1 and IL-6 levels were in accord with the NF-*κ*B levels but opposite to the HO-1 and PPAR*γ* levels. The results collectively demonstrated that the induction of HO-1 expression could suppress TGF-*β*1 and IL-6 secretion from HSCs; the suppressive effects were directly mediated by downregulating NF-*κ*B activity and likely by upregulating PPAR*γ* levels to indirectly affect NF-*κ*B activity.

RETRACTED

In conclusion, HO-1 induction could upregulate PPAR*γ* expression while also directly or indirectly downregulating NF-*κ*B activation in activated HSCs, thus impacting the release of inflammatory cytokines. These pathways represent the protective mechanisms of HO-1 on the liver by inhibiting HSC proliferation and activation, which provides a promising therapeutic strategy for liver fibrosis.

## Figures and Tables

**Figure 1:** Selection for the most appropriate concentrations and incubation periods for Hemin and ZnPP-IX. (a) The effects of the different concentrations of Hemin and ZnPP-IX on HSC-T6 proliferation were assessed by the MTT assay. Hemin suppressed HSC proliferation in a dose-dependent manner, which was significant at 24 hours (*P* < 0.01). Moreover, ZnPP-IX dose-dependently promoted HSC proliferation, which was significant at 24 hours (*P* < 0.05). (b) LDH level in cultured HSC-T6 cells exposed to Hemin or ZnPP-IX. H-A, H-B, and H-C: 6.5, 13, and 26 *μ*g/ml Hemin, respectively; Z-A, Z-B, and Z-C: 3, 6, and 12 *μ*g/ml ZnPP-IX, respectively. There were no significant differences in LDH release from the cells treated with 6.5 and 13 *μ*g/ml Hemin for 12 or 24 hours relative to the control (*P* = 0.83, *P* = 0.128, *P* = 0.553, and *P* = 0.151, respectively). However, LDH release from the cells treated with 6.5 or 13 *μ*g/ml Hemin for 48 hours or with 26 *μ*g/ml Hemin for all time points was notably enhanced compared to that from the normal (*P* < 0.05). For the ZnPP-IX-treated group, the LDH release levels from the cells treated with 12 *μ*g/ml ZnPP-IX for 24 hours and with all concentrations for 48 hours were significantly elevated as compared to those for the normal (*P* < 0.01).

**Figure 2:** HO-1 expression and its effects on HSC proliferation. (a) HO-1 mRNA expression was detected with real-time PCR after the cells were exposed to Hemin or ZnPP-IX. (b) The HO-1 protein level was detected using Western blotting. (c) Effect of HO-1 expression on HSC-T6 cell proliferation. The MTT results for the normal, Hemin-treated, and ZnPP-IX-treated groups were 1.034 ± 0.003, 0.867 ± 0.023, and 1.161 ± 0.015, respectively. ^∗^*P* < 0.01 vs. the normal group; ^▲^*P* < 0.05 vs. the Hemin-treated group.

**Figure 3:** Effects of HO-1 on *α*-SMA expression in HSCs. (a) *α*-SMA protein expression in HSC-T6 cells via Western blot analysis. ^∗^*P* < 0.01 vs. the normal group. ^▲^*P* < 0.01 vs. the Hemin-treated group. (b) *α*-SMA mRNA level in HSC-T6 cells by real-time PCR. ^∗^*P* < 0.01 vs. the normal group; ^▲^*P* < 0.05 vs. the normal group; ^△^*P* < 0.05 vs. the Hemin-treated group. (c) Effects of Hemin or ZnPP-IX on *α*-SMA expression in HSC-T6 cells, as detected by immunocytochemistry (×400).

**Figure 4:** The HA and PIIIP levels in the HSC-T6 supernatant. ^∗^*P* < 0.01 vs. the normal group; ^▲^*P* < 0.05 vs. the normal group; ^△^*P* < 0.01 vs. the Hemin-treated group.

**Figure 5:** Effects of HO-1 on PPAR*γ* and NF-*κ*B expression in HSCs. (a) Effects of HO-1 on PPAR*γ* and NF-*κ*B mRNA expression in HSC-T6 cells. (b) Effects of HO-1 on PPAR*γ* and NF-*κ*B protein expression in HSC-T6 cells. ^∗^*P* < 0.01 vs. the normal group; ^▲^*P* < 0.05 vs. the normal group; ^△^*P* < 0.05 vs. the previous group. (c) The PPAR*γ* level in HSC-T6 cells was examined using immunocytochemistry, and NF-*κ*B p65 subunit expression in HSC-T6 cells was tested with immunofluorescence (×400).

**Figure 6:** Effects of HO-1 on TGF-*β*1 and IL-6 secretion from HSCs. ^∗^*P* < 0.01 vs. the normal group; ^▲^*P* < 0.05 vs. the normal group; ^△^*P* < 0.05 vs. the previous group.

RETRACTED

## Data Availability

The authors confirm that the data supporting the findings of this study are available within the article.

## Abbreviations

HSCs: Hepatic stellate cells
HO-1: Heme oxygenase-1
PPAR*γ*: Peroxisome proliferator-activated receptor-gamma
NF-*κ*B: Nuclear factor-kappa B
ECM: Extracellular matrix
*α*-SMA: *α*-Smooth muscle actin
TNF-*α*: Tumor necrosis factor-*α*
LDH: Lactate dehydrogenase
TGF-*β*1: Transforming growth factor-*β*
IL-6: Interleukin-6
HA: Hyaluronic acid
PCIII: Type III procollagen.

## References

[1] Hernández E., Bucio L., Souza V. (2008). Pentoxifylline downregulates *α* (I) collagen expression by the inhibition of I*κ*b*α* degradation in liver stellate cells. *Cell Biology and Toxicology*.

[2] Zardi E., Navarini L., Sambataro G. (2013). Hepatic PPARs: their role in liver physiology, fibrosis and treatment. *Current Medicinal Chemistry*.

[3] Straus D. S., Pascual G., Li M. (2000). 15-Deoxy-delta 12,14-prostaglandin J_2_ inhibits multiple steps in the NF-kappa B signaling pathway. *Proceedings of the National Academy of Sciences of the United States of America*.

[4] Chung S. W., Kang B. Y., Kim S. H. (2000). Oxidized low density lipoprotein inhibits interleukin-12 production in lipopolysaccharide-activated mouse macrophages via direct interactions between peroxisome proliferator-activated receptor-*γ* and nuclear factor-*κ*B. *The Journal of Biological Chemistry*.

[5] Ryter S. W., Alam J., Choi A. M. (2006). Heme oxygenase-1/carbon monoxide: from basic science to therapeutic applications. *Physiological Reviews*.

[6] Du J., Ren W., Zhang Q. (2020). Heme oxygenase-1 suppresses Wnt signaling pathway in nonalcoholic steatohepatitis-related liver fibrosis. *BioMed Research International*.

[7] Lin C. C., Chiang L. L., Lin C. H. (2007). Transforming growth factor-*β*1 stimulates heme oxygenase-1 expression via the PI3K/Akt and NF-*κ*B pathways in human lung epithelial cells. *European Journal of Pharmacology*.

[8] Kim K. S., Cui X., Lee D. S. (2014). Inhibitory effects of benzaldehyde derivatives from the marine fungus Eurotium sp. SF-5989 on inflammatory mediators via the induction of heme oxygenase-1 in lipopolysaccharide-stimulated RAW264.7 macrophages. *International Journal of Molecular Sciences*.

[9] Ndisang J. F. (2014). Cross-talk between heme oxygenase and peroxisome proliferator-activated receptors in the regulation of physiological functions. *Frontiers in Bioscience*.

[10] Krönke G., Kadl A., Ikonomu E. (2007). Expression of heme oxygenase-1 in human vascular cells is regulated by peroxisome proliferator- activated receptors. *Arteriosclerosis, Thrombosis, and Vascular Biology*.

RETRACTED

[11] Li M., Li Z., Sun X. (2010). Heme oxygenase-1/p21WAF1 mediates peroxisome proliferator-activated receptor-*γ* signaling inhibition of proliferation of rat pulmonary artery smooth muscle cells. *FEBS Journal*.

[12] Yang H., Zhao L. F., Zhao Z. F., Wang Y., Zhao J. J., Zhang L. (2012). Heme oxygenase-1 prevents liver fibrosis in rats by regulating the expression of PPAR*γ* and NF-*κ*B. *World Journal of Gastroenterology*.

[13] Supinski G. S., Callahan L. A. (2006). Hemin prevents cardiac and diaphragm mitochondrial dysfunction in sepsis. *Free Radical Biology & Medicine*.

[14] Liu H., Song D., Lee S. S. (2001). Role of heme oxygenase-carbon monoxide pathway in pathogenesis of cirrhotic cardiomyopathy in the rat. *American Journal of Physiology. Gastrointestinal and Liver Physiology*.

[15] Martasek P., Schwartzman M. L., Goodman A. I., Solangi K. B., Levere R. D., Abraham N. G. (1991). Hemin and L-arginine regulation of blood pressure in spontaneous hypertensive rats. *Journal of the American Society of Nephrology*.

[16] Chen A., Zhang L., Xu J., Tang J. (2002). The antioxidant (-)-epigallocatechin-3-gallate inhibits activated hepatic stellate cell growth and suppresses acetaldehyde-induced gene expression. *The Biochemical Journal*.

[17] Livak K. J., Schmittgen T. D. (2001). Analysis of relative gene expression data using real-time quantitative PCR and the 2^−*ΔΔC*^_T_ method. *Methods*.

[18] Palipoch S., Koomhin P., Punsawad C., Na-Ek P., Sattayakhom A., Suwannalert P. (2016). Heme oxygenase-1 alleviates alcoholic liver steatosis: histopathological study. *Journal of Toxicologic Pathology*.

[19] Tang J., Li C. M., Li L., Wu J., Wang G. L. (2016). Changes in expression and production of heme oxygenase-1 in rats with acute liver injury induced by lipopolysaccharide. *The Journal of Toxicological Sciences*.

[20] Bakhautdin B., Das D., Mandal P. (2014). Protective role of HO-1 and carbon monoxide in ethanol-induced hepatocyte cell death and liver injury in mice. *Journal of Hepatology*.

[21] Vogel S., Piantedosi R., Frank J. (2000). An immortalized rat liver stellate cell line (HSC-T6): a new cell model for the study of retinoid metabolism in vitro. *Journal of Lipid Research*.

[22] Zhang F., Kong D., Lu Y., Zheng S. (2013). Peroxisome proliferator-activated receptor-*γ* as a therapeutic target for hepatic fibrosis: from bench to bedside. *Cellular and Molecular Life Sciences*.

[23] Guo Y. T., Leng X. S., Li T. (2005). Effect of ligand of peroxisome proliferator-activated receptor gamma on the biological characters of hepatic stellate cells. *World Journal of Gastroenterology*.

RETRACTED

[24] Zong L., Qu Y., Xu M. Y., Dong Y. W., Lu L. G. (2013). 18*α*-Glycyrrhetinic acid extracted fromGlycyrrhiza radixinhibits proliferation and promotes apoptosis of the hepatic stellate cell line. *Journal of Digestive Diseases*.

[25] Yeh C. H., Chen T. P., Wang Y. C., Lin Y. M., Lin P. J. (2009). HO-1 activation can attenuate cardiomyocytic apoptosis *via* inhibition of NF- *κ*B and AP-1 translocation following cardiac global ischemia and reperfusion. *The Journal of Surgical Research*.

[26] Liu Z., Ai Y., Zhang L. (2009). Effect of hemin on severe acute pancreatitis-associated lung injury in rats and its mechanism. *Zhong nan da xue xue bao. Yi xue ban= Journal of Central South University. Medical Sciences*.

[27] Lee I. T., Luo S. F., Lee C. W. (2009). Overexpression of HO-1 protects against TNF-*α*-mediated airway inflammation by down-regulation of TNFR1-dependent oxidative stress. *The American Journal of Pathology*.

[28] Zhao C., Chen W., Yang L., Chen L., Stimpson S. A., Diehl A. M. (2006). PPAR*γ* agonists prevent TGF*β*1/Smad3-signaling in human hepatic stellate cells. *Biochemical and Biophysical Research Communications*.

[29] Elsharkawy A. M., Mann D. A. (2007). Nuclear factor-*κ*B and the hepatic inflammation-fibrosis-cancer axis. *Hepatology*.

